# Posaconazole Exhibits *In Vitro* and *In Vivo* Synergistic Antifungal Activity with Caspofungin or FK506 against *Candida albicans*

**DOI:** 10.1371/journal.pone.0057672

**Published:** 2013-03-05

**Authors:** Ying-Lien Chen, Virginia N. Lehman, Anna F. Averette, John R. Perfect, Joseph Heitman

**Affiliations:** 1 Department of Molecular Genetics and Microbiology, Duke University Medical Center, Durham, North Carolina, United States of America; 2 Department of Plant Pathology and Microbiology, National Taiwan University, Taipei, Taiwan; 3 Department of Biomedical Engineering, Duke University, Durham, North Carolina, United States of America; 4 Department of Medicine, Duke University Medical Center, Durham, North Carolina, United States of America; Yonsei University, Republic of Korea

## Abstract

The object of this study was to test whether posaconazole, a broad-spectrum antifungal agent inhibiting ergosterol biosynthesis, exhibits synergy with the β-1,3 glucan synthase inhibitor caspofungin or the calcineurin inhibitor FK506 against the human fungal pathogen *Candida albicans*. Although current drug treatments for *Candida* infection are often efficacious, the available antifungal armamentarium may not be keeping pace with the increasing incidence of drug resistant strains. The development of drug combinations or novel antifungal drugs to address emerging drug resistance is therefore of general importance. Combination drug therapies are employed to treat patients with HIV, cancer, or tuberculosis, and has considerable promise in the treatment of fungal infections like cryptococcal meningitis and *C. albicans* infections. Our studies reported here demonstrate that posaconazole exhibits *in vitro* synergy with caspofungin or FK506 against drug susceptible or resistant *C. albicans* strains. Furthermore, these combinations also show *in vivo* synergy against *C. albicans* strain SC5314 and its derived echinocandin-resistant mutants, which harbor an S645Y mutation in the CaFks1 β-1,3 glucan synthase drug target, suggesting potential therapeutic applicability for these combinations in the future.

## Introduction

*Candida albicans* is the leading *Candida* species causing bloodstream infections (candidemia), oral thrush, and vaginal yeast infections [1], [2]. Candidemia often results in a high mortality rate (>30%), particularly if appropriate antifungal drug treatments are delayed [3]. The increase of *Candida* infection is, in part, due to rising numbers of immunocompromised patients and widespread use of broad spectrum antibiotics. Azoles, echinocandins, amphotericin B, and flucytosine are current antifungal drugs for treating *Candida* infections. However, the implementation of these and other antifungal drugs has not kept pace with the increased incidence of drug-resistance. Therefore, either a combination of current drugs or development of novel antifungal drugs will be important for present and future therapy. Posaconazole inhibits lanosterol 14α-demethylase required for ergosterol biosynthesis and is the most recently approved triazole with broad spectrum activity against *Candida*, *Cryptococcus*, *Aspergillus*, zygomycetes, dermatophytes, and other fungal pathogens [4]. Caspofungin inhibits β-1,3 glucan synthesis and represents the newest class of antifungal drugs, with an excellent safety profile [5]. FK506 (tacrolimus) is an immunosuppressant for organ transplant that targets both mammalian and fungal calcineurins [6], [7].

Drug-resistant *C. albicans* strains have been frequently isolated from patients [8]. For example, White et al. reported a series of 17 sequential isolates associated with the emergence of azole resistance in an HIV-infected patient [9]. Furthermore, the azole resistance of the 17 isolates was correlated with increased mRNA levels of the *ERG11*, *CDR1*, and *MDR1* genes in *C. albicans* [10]. Garcia-Effron et al. isolated *C. albicans* echinocandin resistant strains associated with β-1,3 glucan synthase *FKS1* mutations [11]. These echinocandin resistant strains have a breakpoint at 2 µg/ml for caspofungin, and 0.5 µg/ml for micafungin and anidulafungin. However, approaches to treat these infections caused by drug resistant isolates are lacking or patients must receive the toxic polyene antifungals.

Combination therapy, also known as cocktail therapy or Highly Active Antiretroviral Therapy (HAART), was first used to inhibit HIV virus replication via multiple mechanisms [12], [13], [14], and now is one of the most successful approaches to combating infectious diseases. Therefore, it is possible that drug combinations with different mechanisms of action such as posaconazole, caspofungin, and FK506 can be deployed to manage *C. albicans* infection. It has been demonstrated that posaconazole alone at a dose of 2.5 mg/kg can reduce *C. albicans* colonization in the kidney tissues in an immunocompromised mouse model [15]. However, whether posaconazole exhibits *in vivo* synergy with other antifungal drugs against *C. albicans* drug-susceptible or drug-resistant isolates was unclear.

In this study we set out to test the potential efficacy of posaconazole when combined with either caspofungin or FK506 in treating *C. albicans* infection in a murine systemic infection model. We found that posaconazole exhibits *in vitro* synergistic antifungal activity with either caspofungin or FK506 against drug susceptible or resistant clinical *C. albicans* isolates. Although these combinations were not found to exhibit *in vivo* synergistic activity against several clinical drug-resistant isolates, they were efficacious against both *C. albicans* SC5314-derived echinocandin-resistant mutant YC734 and its wild-type parental isolate SC5314.

## Materials and Methods

### *C. albians* Strains used in this Study

*C. albicans* strains used in this study are listed in Table 1. In brief, four clinical echinocandin-resistant isolates 89, 177, 194 and 205 with different mutations in the Fks1 protein [11] were chosen to determine the efficacy of drug combination against echinocandin-resistant isolates. Meanwhile, three clinical isolates representing #1 (2–76), #9 (2–86), and #17 (12–99) of a series of 17 sequential isolates were chosen, and which are associated with the emergence of fluconazole resistance and increased expression levels of *ERG11*, *CDR1* and *MDR1* in an HIV-infected patient [9], [10]. Due to step-wise increased fluconazole resistance, isolates 2–76 and 2–86 are fluconazole-susceptible, while 12–99 is a fluconazole-resistant isolate [9]. Interestingly, these isolates were susceptible to posaconazole although 12–99 has an MIC_50_ ∼10 fold higher than the 2–76 or 2–86 isolate (Table 2). In addition, we generated SC5314-derived genetically engineered echinocandin resistant strains YC734 and YC736 with an S645Y mutation in the *C. albicans* Fks1 protein (refer to the section on strain construction for details).

**Table 1:** *Candida albicans* strains used in this study.

Strain	Description	Background	Reference
SC5314	Prototrophic wild-type SC5314	Clinical isolate	[46]
89	Echinocandin resistant (Fks1 S645Y)	Clinical isolate	[11]
177	Echinocandin resistant (Fks1 F641S)	Clinical isolate	[11]
194	Echinocandin resistant (Fks1 S645F)	Clinical isolate	[11]
205	Echinocandin resistant (Fks1 S645P)	Clinical isolate	[11]
2–76	1/17 azole resistant series strain	Clinical isolate	[9]
2–86	9/17 azole resistant series strain	Clinical isolate	[9]
12–99	17/17 azole resistant series strain	Clinical isolate	[9]
YC734	Fks1 S645Y (independent isolate #1)	SC5314	This study
YC736	Fks1 S645Y (independent isolate #2)	SC5314	This study

**Table 2:** Synergistic antifungal activity between posaconazole and caspofungin or FK506 against *C. albicans* drug susceptible or resistant strains.

C. albicans	PSC		CSF		FK506		MIC_100_ combined		*FIC index	
	MIC_50_	MIC_100_	MIC_50_	MIC_100_	MIC_50_	MIC_100_	(PSC,CSF)	(PSC,FK506)	PSC+CSF	PSC+FK506
SC5314#	0.03	>16	0.06	0.25	>16	>16	4,0.03	0.06,0.25	0.25	0.01
89	0.25	>16	2	>16	1	>16	0.06,16	1,0.25	0.5	0.04
177	0.03	>16	2	>16	>16	>16	0.03,16	0.25,8	0.5	0.26
205	0.25	>16	>16	>16	2	>16	0.06,16	0.25,4	0.5	0.13
194	0.5	>16	>16	>16	>16	>16	0.03,16	0.13,2	0.5	0.07
2–76	<0.03	>16	0.5	>16	>16	>16	0.03,8	0.03,1	0.25	0.03
2–86	<0.03	>16	0.25	>16	>16	>16	0.25,4	0.06,2	0.13	0.06
12–99	0.13	>16	0.25	>16	>16	>16	0.25,4	0.13,0.5	0.13	0.02
YC734	0.03	>16	2	>16	>16	>16	0.13,4	0.06,0.5	0.13	0.02
YC736	0.03	>16	2	>16	>16	>16	0.5,4	0.06,0.25	0.14	0.01

# Orange highlighting color indicates wild-type and its derived mutants, while yellow and green highlighting colors represent echinocandin resistant and 3 (#1, #9, #17) out of 17 azole resistant isolates from the strain series, respectively.

* Formula of FIC index:

[(MIC_100_ of drug A in combination)/(MIC_100_ of drug A alone)]+[(MIC_100_ of drug B in combination)/(MIC_100_ of drug B alone)].

FIC≤0.5 (Synergy); FIC >4 (Antagonism); FIC >0.5 but ≤4 (no interaction).

### Determination of Minimum and Fractional Inhibitory Concentration Indices

We determined minimum inhibitory concentrations (MIC) by the Clinical and Laboratory Standards Institute (CLSI) protocol M27-A3, while fractional inhibitory concentration (drug interaction) was assessed via checkerboard titration assays. Testing was done in RPMI-1640, buffered to pH 7.0 with 0.165 M MOPS. Yeast strains were grown in YPD medium overnight, incubated at 30°C with shaking, and washed twice with dH_2_O. The OD_600_ was measured and each strain was diluted to 1 OD_600_/ml. This inoculum was then diluted to 0.0005 OD_600_/ml in RPMI-1640. 98 µl of the strain culture was added to each well in a 96 well plate format. 2 µl of serially diluted drugs were added to the wells, yielding a total volume of 100 µl per well. Posaconazole was added across the plate with the highest concentration in the left well and the lowest concentration in the right well. Posaconazole concentrations ranged from 0.03–16 µg/ml. Either caspofungin or FK506 was added from top to bottom, with the highest concentration in the top row and the lowest concentration in the bottom row. Caspofungin and FK506 concentrations ranged from 0.25–16 µg/ml. This strategy allowed for 70 different drug concentrations to be tested on one plate. The plates were incubated for ∼48 hours at 30°C, and then the OD_600_ of each plate was read. The *in vitro* drug interaction studies were performed at least twice. The minimum inhibitory concentration (MIC_100_) of both drugs, either alone or in combination, was defined as the lowest concentration of each drug which resulted in total inhibition of visible fungal growth [16] and produced a 99.9% of inhibition based on spectrophotometric determination at OD_600_ when compared to the control well. Meanwhile, MIC_100_ was found to be equivalent to the minimum fungicidal concentration (MFC) for *C. albicans* isolates [16]. The fractional inhibitory concentration (FIC) was calculated by: (MIC_combined_ drug A/MIC_alone_ drug A)+(MIC_combined_ drug B/MIC_alone_ drug B). A FIC index of ≤0.5 indicates synergy, >4.0 indicates antagonism, and an index between 0.5 and 4 indicates no interaction [17]. For calculation purposes, an MIC >16 was assumed to be 32.

### Ethics Statement

Animals studies were conducted in the Division of Laboratory Animal Resources (DLAR) facilities at Duke University Medical Center (DUMC) in good practice as defined by the United States Animal Welfare Act and in full compliance with the guidelines of the DUMC Institutional Animal Care and Use Committee (IACUC). The vertebrate animal experiments were reviewed and approved by the DUMC IACUC under protocol number A165-11-06.

### Mouse Infection and Drug Treatments

Four- to five-week-old male CD1 mice (Jackson Laboratory, ∼30 g) were used in this study. For infection, *C. albicans* strains were cultured in YPD broth overnight at 30°C and washed twice with sterile PBS. Cells were counted with a hemocytometer, and resuspended in sterile PBS at 5×10^6^ cells per ml. Dilutions of the cells were plated onto YPD and incubated at 30°C for 48 hr to determine CFU and viability. Groups of 5 or 10 mice were inoculated with *C. albicans* via tail-vein injection of 10^6^ cells (in 200 µl). The *in vivo* dosing regimens including dose level, dosing interval, and treatment duration were chosen from previous work in the literature [15], [18], [19], [20] and from our prior knowledge of pilot experiments for a susceptible *C. albicans* SC5314 strain. Posaconazole (NOXAFIL, Merck & Co.) was diluted with PBS and administered via oral gavage (Roboz Cat#FN-7920; 22 gauge), while placebo PBS, caspofungin (provided by Merck), and FK506 (provided by Astellas) were administered via the intraperitoneal route (in 100 µl) after 4, 24, 48, and 72 hr following *Candida* infection. The conditions of the mice were monitored 1 to 2 times daily, and moribund mice were euthanized with CO_2_. Kaplan-Meier survival curves were generated with Prism 5.03 (GraphPad software, La Jolla, CA, USA), and *P* values were evaluated by a Log-rank (Mantel-Cox) test. A *P* value of <0.05 was considered significant.

### Construction of the *FKS1-1* Mutants

The *FKS1-1* mutant strains were constructed by direct transformation of *C. albicans* strain SC5314 by electroporation with 10 µg of a mutagenic 90-mer synthetic oligonucleotide JC583 (CCTTGCCAAATTGGTTGAATCTTATTTCTTCTTGACATTGTATTTGAGAGATCCTATTAGAAACTTGTCGACCATGACAATGAGATGTGT) [21], [22]. JC583 is identical to nucleotides 1893 to 1982 of the sense strand of the *FKS1* ORF (orf19.2929) except at the underlined nucleotides, which introduce a C1934A (S645Y) and A1938G (silent marker; only changed in third nucleotide of the codon, but not amino acid in order to rule out spontaneous S645Y mutations occurring during selection). The PflFI site (GACnnnGTC) present in the wild-type allele was eliminated by introduction of the C1934A mutation. Transformants were selected on YPD plates containing 1 µg/ml caspofungin. Two independent echinocandin-resistant strains (YC734, YC736) derived from different transformations were obtained. These strains were confirmed by PCR of the *FKS1* locus with primers JC584 (GCATCACAAACATTTACTGCC) and JC585 (CGTGGTAGCTAAAATCTTGG) and subsequent DNA sequencing (Eton Bioscience Inc.). The JC584/JC585 PCR products were also treated with ExoSAP-it and further digested with the restriction enzyme PflFI, which recognizes the GACnnnGTC sequence that is present in wild-type (SC5314) but not in the isogenic *FKS1-1* mutants (YC734, YC736) and clinical isolate 89. The silent A1938G mutation was confirmed by DNA sequencing and digestion with restriction enzyme MseI.

## Results

### Posaconazole Exhibits Synergistic Antifungal Activity with Caspofungin *in vitro* and *in vivo* Against *C. albicans* SC5314

Two different antifungal drugs with distinct mechanisms for targeting pathogens can potentially exhibit synergistic antifungal activity [23], [24]. Posaconazole has been demonstrated to exhibit *in vitro* synergistic antifungal activity with caspofungin against human fungal pathogens, including *C. albicans* [25], [26], *C. glabrata* [27] and *A. fumigatus* [28]. Although an *in vivo* synergistic antifungal activity between posaconazole and caspofungin has been shown for *A. fumigatus* infection [28], it has not yet been similarly demonstrated for *C. albicans*. Here, we demonstrate that posaconazole exhibits *in vitro* synergistic antifungal activity with caspofungin against not only the *C. albicans* strain SC5314, but also fluconazole- or echinocandin-resistant isolates [Fractional Inhibitory Concentration (FIC)≤0.5; Table 2]. In animal infections with drug therapeutic experiments, we demonstrate that posaconazole (orally administered) alone at 2 mg/kg has therapeutic antifungal activity against *C. albicans* strain SC5314 (*P* = 0.002; log-rank test, Figure 1A) and the fluconazole resistant isolate 12–99 (*P* = 0.005; Figure 1B); while caspofungin (intraperitoneal administered) alone at 0.1 mg/kg exhibits therapeutic activity against *C. albicans* SC5314 (*P* = 0.002; Figure 1A), 12–99 (*P* = 0.002; Figure 1B), and the echinocandin-resistant isolate 89 (*P* = 0.03; Figure 1C). In combination drug therapy, the animals infected with *C. albicans* SC5314 and treated with posaconazole at 2 mg/kg and caspofungin at 0.1 mg/kg survived longer than infected groups treated with posaconazole (2 mg/kg; *P* = 0.002) or caspofungin (0.1 mg/kg; *P* = 0.03) monotherapy (Figure 1A). However, the posaconazole-caspofungin drug combination therapy did not show *in vivo* synergy against the drug resistant isolates 12–99 (fluconazole) or 89 (echinocandin) (Figure 1B and 1C).

**Figure 1:** Efficacy of posaconazole and caspofungin against *C. albicans* infection. Five male CD1 mice (4–5 weeks-old) per group were infected with 10^6^ cells of *C. albicans* SC5314, azole-resistant isolate 12–99, or echinocandin-resistant isolate 89, followed by treatment with placebo (PBS), posaconazole (PSC; 2 mg/kg), caspofungin (CSF; 0.1 mg/kg), or PSC (2 mg/kg) plus CSF (0.1 mg/kg). The PSC was administered via oral gavage, while PBS and CSF were administered via intraperitoneal injection at 4, 24, 48, and 72 hr post infection. Survival of the animals was monitored for up to 35 days.

### Posaconazole Exhibits Synergistic Antifungal Activity with FK506 *in vitro* and *in vivo* Against *C. albicans* SC5314

Fluconazole has been demonstrated to exhibit *in vitro* synergistic antifungal activity with the immunosuppressant FK506 or cyclosporin A against *Candida* species [29], [30], [31], [32], [33], [34], [35] but this had not yet been reported for posaconazole. Furthermore, it was unclear if posaconazole exhibits the same *in vitro* and *in vivo* synergy with FK506 against *C. albicans* infection. Here, we demonstrate that posaconazole exhibits *in vitro* synergistic antifungal activity with FK506 against not only the *C. albicans* SC5314 type strain, but also with the clinical azole- or echinocandin-resistant isolates (FIC<0.5, Table 2). For monotherapy with either posaconazole or FK506, we found that posaconazole at 0.5 mg/kg exhibited therapeutic activity against *C. albicans* SC5314, but not against fluconazole-resistant isolate 12–99 (2 mg/kg is required for therapeutic response; Figure 1B) or the echinocandin-resistant isolate 89 (Figures 2B and 2C). On the other hand, FK506 at 0.5 mg/kg had no therapeutic activity against *C. albicans* SC5314 or the drug-resistant strains (Figure 2). For the combination therapy of posaconazole plus FK506, we found that posaconazole exhibits modest *in vivo* synergy with FK506 against *C. albicans* SC5314 (*P*≤0.02; Figure 2A), but no apparent synergy against the fluconazole-resistant 12–99 or echinocandin-resistant 89 isolates (Figures 2B and 2C).

**Figure 2:** Efficacy of posaconazole and FK506 against *C. albicans* infection. Ten male CD1 mice (4–5 weeks-old) per group were infected with 10^6^ cells of *C. albicans* SC5314, azole-resistant isolate 12–99, or echinocandin-resistant isolate 89, followed by treatment with placebo (PBS), posaconazole (PSC; 0.5 mg/kg), FK506 (0.5 mg/kg), or PSC (0.5 mg/kg) plus FK506 (0.5 mg/kg). The PSC was administered via oral gavage, while PBS and FK506 were administered via intraperitoneal injection at 4, 24, 48, and 72 hr post inoculation. Survival of the animals was monitored for up to 18 days.

### Serine 645 of the CaFks1 Protein is Essential for Echinocandin, but not Azole Resistance, in *C. albicans*

Our data show that the clinical *C. albicans* echinocandin resistant isolate 89, which has an S645Y mutation in the CaFks1 protein [11], exhibits caspofungin resistance (MIC_100_>16 µg/ml), and an 8-fold reduced susceptibility to posaconazole (MIC_50_ = 0.25 µg/ml) compared with SC5314 (MIC_50_ = 0.03 µg/ml). Because echinocandin resistant isolate 89 and SC5314 are both clinically derived, but not isogenic strains, and isolate 89 has reduced azole susceptibility along with its echinocandin resistance, the contribution of echinocandin resistance and reduced posaconazole susceptibility of isolate 89 may be due to certain strain differences, but not strictly attributable to the S645Y mutation for echinocandin resistance. To test this possibility, we introduced an S645Y mutation in the CaFks1 protein of *C. albicans* SC5314 via mutagenic oligonucleotide transformation. Two independent mutants (YC734 and YC736) with the C1934A (S645Y) mutation in the *CaFKS1* gene were derived from different transformations (Table 1). The C1934A (S645Y) and A1938G mutations of the *CaFKS1* sequences of the wild-type SC5314, YC734, YC736, and 89 strains were confirmed by DNA sequencing (Figure 3A), and two restriction enzymes (PflFI and MseI) that distinguish C1934A (S645Y) (Figure 3B) and the A1938G silent mutation (Figure 3C) from wild-type DNA sequences, respectively.

**Figure 3:** Confirmation of *C. albicans FKS1-1* mutants with the S645Y mutation. (**A**) Genomic DNA from SC5314 (wild-type), the *FKS1-1* mutants (YC734 and YC736), and isolate 89 were PCR amplified with primers JC584/JC585 to detect a 410 bp (1810∼2220) product of the *CaFKS1* gene, and then sequenced with primer JC584. Nucleotide 1934 of the *CaFKS1* gene is labeled green. The C1934A mutation is present in *FKS1-1* mutants derived from SC5314 and in the clinical isolate 89, but absent in SC5314. Nucleotide 1938 of the *CaFKS1* gene is labeled purple. An A1938G silent mutation is present in the *FKS1-1* mutants, but not in SC5314 or isolate 89. (**B**)**&**(**C**) The 410 bp PCR product of the *CaFKS1* gene was amplified from genomic DNA from SC5314, *FKS1-1* mutants (YC734 and YC736), and isolate 89, and digested with PflFI (**B**) or MseI (**C**) to confirm the C1934A or A1938G mutations are present and to confirm the mutations occurred in both alleles of the gene.

We found that YC734 and YC736 strains with the S645Y amino acid change are tolerant to 1 µg/ml of caspofungin, micafungin, or anidulafungin, while their parent strain SC5314 is susceptible to all three at this concentration (Figure 4A). These results are similar to the echinocandin resistant isolate 89 (Figure 4A), suggesting that the serine amino acid at position 645 of the CaFks1 protein is essential for echinocandin sensitivity. We further found that the echinocandin-resistant isolate 89 is tolerant to multiple azoles (including posaconazole, fluconazole, and ketoconazole) compared with the SC5314, YC734, and YC736 strains (Figure 4B). These results indicate that 1) different clinical isolates can exhibit distinct azole tolerance profiles; 2) isolate 89 may harbor additional mutation(s) altering drug pumps or multi-drug resistance or *ERG11* genes that contribute to azole tolerance, and that we might not be simply measuring echinocandin-resistance *in vivo* when combination therapy is given.

**Figure 4:** *In vitro* phenotypes and the *in vivo* efficacy of posaconazole combined with either caspofungin or FK506 against *C. albicans FKS1-1* mutant. Cells were grown overnight in YPD at 30°C, 5-fold serially diluted, spotted onto YPD medium containing an echinocandin (**A**) or an azole (**B**) at the concentrations indicated, and incubated at 37°C for 48 hr. The efficacy of posaconazole (2 mg/kg) and caspofungin (0.1 mg/kg) (**C**) or posaconazole (0.5 mg/kg) and FK506 (0.5 mg/kg) (**D**) against the *C. albicans FKS1-1* mutant (YC734). The experimental procedures are similar to those described in the legend to Figure 1, except that the survival of the animals was monitored for up to 21 days.

### Posaconazole Exhibits *in vivo* Synergy with Caspofungin or FK506 against Echinocandin-resistant Mutant Generated from *C. albicans* SC5314

Because the clinical echinocandin-resistant isolate 89 exhibits reduced susceptibility to posaconazole compared with the *C. albicans* SC5314 isolate, this difference might have affected the *in vitro* and *in vivo* interaction between posaconazole and caspofungin or FK506 against the 89 and SC5314 isolates. To test this hypothesis, we determined the *in vitro* and *in vivo* efficacy of posaconazole and caspofungin or FK506 against echinocandin-resistant mutants (YC734 and YC736) generated from the isogenic SC5314 isolate. Our *in vitro* analyses show that, similar to isolate 89, YC734 and YC736 are tolerant to echinocandins, and exhibit similar posaconazole susceptibility profiles to SC5314, but not to isolate 89 (Figure 4 and Table 2). In checkerboard assays, we found that posaconazole exhibits *in vitro* synergy with caspofungin or FK506 against the YC734 and YC736 mutants (FIC<0.5), and the isolate 89 (FIC≤0.5; Table 2). Furthermore, our *in vivo* efficacy experiments demonstrated that either the posaconazole-caspofungin or the posaconazole-FK506 combination therapy exhibited synergistic antifungal activity (*P*<0.05) against echinocandin-resistant strain YC734, an isogenic derivative of SC5314 (Figures 4C and 4D).

## Discussion

Our studies demonstrate that posaconazole exhibits synergistic antifungal activity with caspofungin *in vitro* and *in vivo* against the wild-type *C. albicans* isolate SC5314 (Table 2 and Figure 1), suggesting both posaconazole and caspofungin can be effectively combined to treat candidiasis in the murine model of systemic infection, which could possibly lead to better treatment options for patients such as those with endocarditis. While *in vitro* synergy was seen across the various strains, the *in vivo* synergy between posaconazole and caspofungin is not evident against the fluconazole-resistant 12–99 or the echinocandin-resistant 89 isolates. This is possibly due to different drug-resistance profiles and/or strain backgrounds between SC5314 and these wild type drug-resistant isolates 12–99 or 89, and demonstrates how variable but important synergy studies can be for *in vivo* experiments.

Graybill et al. reported that the addition of caspofungin to fluconazole does not exhibit *in vivo* synergistic antifungal activity in murine candidiasis [36]. On the other hand, previous studies demonstrated that posaconazole and caspofungin exhibited synergistic antifungal activity without evidence of antagonism against *C. glabrata* (*in vitro*) and *A. fumigatus* (*in vitro* and in a murine aspergillosis model) [27], [28]. Therefore, these studies support a clinical trial or occasional empirical use of these combinations because there is no antagonism found between fluconazole/posaconazole and caspofungin. Our studies have similarly found no antagonism (*in vitro* or *in vivo*) between posaconazole and caspofungin against both *C. albicans* SC5314, and drug-resistant clinical isolates. Interestingly, we specifically found that posaconazole exhibits *in vivo* synergy with caspofungin (Figure 1), which supports the hypothesis that these two drug classes with different targets are able to therapeutically synergize. The reported differences in the *in vivo* synergy profiles between posaconazole/caspofungin and fluconazole/caspofungin combinations may be due to 1) structural and spectrum differences between posaconazole and fluconazole [37], 2) differences in experimental protocols between labs, and/or 3) differences in *C. albicans* strains and/or mouse backgrounds. Previous studies had reported that patients with azole-resistant *C*. *albicans* infections can be cured with posaconazole [38], indicating a potential advantage of posaconazole against azole-resistant isolates. This feature was also supported by our finding that posaconazole treatment at a dose of 2 mg/kg (but not 0.5 mg/kg) exhibited therapeutic activity against the azole (especially fluconazole)-resistant isolate 12–99 (Figures 1B and 2B). The reason that the posaconazole-caspofungin drug combination therapy was only efficacious against the wild-type SC5314 strain, but not to fluconazole-resistant isolate 12–99 or echinocandin-resistant isolate 89, might be due to 1) insufficient doses administered to the drug-resistant isolates compared with the wild-type, or 2) high inoculum (10^6^ cells) of drug-resistant isolate used might overwhelm the antifungal activity, or 3) cross resistance/tolerance of isolate 12–99 to caspofungin (Table 2 and data not shown) or isolate 89 to azoles (Figure 4B). For example, Schuetzer-Muehlbauer et al. demonstrated that high levels of *C. albicans* Cdr2 expression confer cross resistance to multiple antifungal drugs attributable to increased drug efflux [39].

Posaconazole has been demonstrated to show in *vitro* synergistic antifungal activity with a calcineurin inhibitor (FK506 or cyclosporin A) against zygomycetes. For example, Dannaoui et al. found that posaconazole has *in vitro* synergy with cyclosporin A against *Mycocladus corymbiferus* [40], while Narreddy et al. showed that posaconazole exhibits *in vitro* synergy with cyclosporin A or FK506 against *Myocladus corymbifera*, *Cunninghamella bertholletiae*, or *Apophysomyces elegans* [41]. Although the data of *in vivo* synergy between posaconazole and a calcineurin inhibitor against *C. albicans* are lacking, Lewis et al. recently reported that posaconazole and FK506 show *in vivo* synergy against *Rhizopus oryzae* in an experimental model of mucormycosis [42]. Furthermore, Marchetti et al. reported that fluconazole exhibits synergy with cyclosporin A against experimental endocarditis due to *C. albicans* [43]. Our data here showed that posaconazole exhibits synergy with FK506 against the *C. albicans* SC5314 strain *in vitro* and *in vivo*. However, posaconazole only exhibits *in vitro* and not *in vivo* synergy with FK506 against the drug-resistant clinical isolates 12–99 or 89 (Table 2; Figure 2). It is evident that posaconazole can be synergistic with FK506 *in vitro* against clinical drug susceptible or resistant *C. albicans* isolates (FIC<0.5; Table 2). The reason that posaconazole only exhibits modest *in vivo* synergistic antifungal activity with FK506 against *C. albicans* SC5314 or none against the drug-resistant 12–99 or 89 isolates may be attributable to immunosuppression by FK506 in the *in vivo* setting in addition to its antifungal activity. Another potential issue is that *in vivo* drug-drug interactions between posaconazole and FK506 could result in the presence of host levels of either drug that can only inhibit drug-susceptible SC5314, but not drug-resistant isolates. Previous studies have shown that posaconazole can inhibit FK506 metabolism by cytochrome P450 (CYP3A4) in cystic fibrosis lung transplant patients to result in ∼3-fold increased levels of FK506 [44], [45]. We attempted to determine if this is the case in our animal model by analyzing the pharmacokinetics of FK506 levels in mouse blood by an LC-MS/MS method. However, in our murine model we did not observe increased blood levels of FK506 when combined with posaconazole (data not shown). This finding may be due to the difficulty of tracing the dynamic changes of blood FK506 levels during our experimental protocols. Another possible explanation for the absence of *in vivo* synergistic antifungal activity between posaconazole and FK506 against two clinical isolates 12–99 and 89 compared with the SC5314 isolate may be attributable to different strain backgrounds and their specific drug-resistance profiles among these isolates.

In summary, we demonstrate that posaconazole exhibits *in vitro* synergy with caspofungin or FK506 against the *C. albicans* isolates tested (Table 2). Furthermore, we show that posaconazole exhibits *in vivo* synergy with caspofungin or FK506 against *C. albicans* strain SC5314, a standard wild type isolate, and a derived echinocandin-resistant mutant, YC734, of this strain. Overall, the combination of posaconazole and caspofungin or FK506 has potentially beneficial combined activity, and no apparent deleterious effects were found within host animals infected with *C. albicans*. These *in vitro* and *in vivo* findings clearly support the potential for combination in a clinical trial to test for improvements in therapeutic endpoints in these fragile patients with invasive candidiasis.
